This article has been retracted.

# Carveol Promotes Nrf2 Contribution in Depressive Disorders through an Anti-inflammatory Mechanism

**DOI:** 10.1155/2022/4509204

**Published:** 2022-03-07

**Authors:** Asmaa Jan Muhammad, Liangliang Hao, Lina Tariq Al Kury, Najeeb Ur Rehman, Arooj Mohsin Alvi, Haroon Badshah, Ikram Ullah, Fawad Ali Shah, Shupeng Li

**Affiliations:** ^1^Riphah Institute of Pharmaceutical Sciences, Riphah International University, Islamabad, Pakistan; ^2^Hospital of Chengdu University of Traditional Chinese Medicine, China; ^3^College of Natural and Health Sciences, Zayed University, Abu Dhabi 49153, UAE; ^4^Department of Pharmacology and Toxicology, College of Pharmacy, Prince Sattam Bin Abdulaziz University, Al-Kharj, Saudi Arabia; ^5^Department of Pharmacy, Abdul Wali Khan University Mardan, Pakistan; ^6^Center for Interdisciplinary Research in Basic Sciences, International Islamic University, Islamabad, Pakistan; ^7^State Key Laboratory of Oncogenomics, School of Chemical Biology and Biotechnology, Shenzhen Graduate School, Peking University, Shenzhen 518000, China

## Abstract

Major depressive disorder (MDD) is a progressive deteriorating mental state with a feeling of worthlessness and frequent mood swings. Several studies reported the favorable effects of natural drug substances on MMD associated oxidative stress and neuroinflammation. The present study is attempted to examine whether carveol could affect lipopolysaccharide- (LPS-) induced depression, and if so, how nuclear factor E2-related factor (Nrf2) contributed to the neuroprotective effects of carveol mechanistically. Two experimental cohorts were used using the SD rats: first to evaluate the promising dose of carveol (whether 20 mg/kg or 50 mg/kg) and secondly to determine the effect of carveol on Nrf2-mediated antidepression. Significant neuronal alterations were noticed in the cortex and hippocampus regions in the LPS-treated group, accompanied by elevated inflammatory cytokine levels such as tumor necrosis factor-alpha (TNF-*α*), cyclooxygenase (COX-2), and c-Jun N-terminal kinase (p-JNK). Moreover, amassing of free radicals exacerbated lipid peroxidase (LPO) and oxidative stress with a limited antioxidant capacity. Carveol (20 mg/kg) significantly ameliorated these detrimental effects by promoting the antioxidant Nrf2 gene and protein, which critically regulate the downstream antioxidant and anti-inflammatory pathway. To further elaborate our hypothesis, we employed all-trans retinoic acid (ATRA), an Nrf2 inhibitor, and we found that ATRA exaggerated LPS-induced depressive-like effects associated with elevated neuroinflammatory markers. Our results demonstrated that carveol (20 mg/kg) could activate the endogenous antioxidant Nrf2, which regulates the downstream antioxidant signaling pathway, eventually leading to amelioration of LPS-induced neuroinflammation and neurodegeneration.

## 1. Introduction

Depressive disorders like major depression or MDD are the leading human problem with multifactorial abnormalities ranging from mood, emotion, and cognitive deficits along with recurrent thoughts of suicide [1, 2]. Depression is increasingly becoming a social and economic problem that costs billions of dollars [3], and up to 60% of suicidal cases could be linked to depressive-like symptoms [4]. Although, depression has been declared as a major contributor to the total burden of world diseases by WHO [5], very little is known about the exact etiological cause and underlying pathophysiology. Moreover, several conditions such as stress exposure, metabolic and hormonal disorders, and drug addiction can precipitate the symptoms. Serotonin and/or norepinephrine-based drugs are extensively used so far, but the effectiveness of such antidepressant drugs is shrinking due to the unpredictable responses and their low recovery ratio. Therefore, looking into the risk-benefit ratio, subsequent alternatives are the demand of the day [6]. Furthermore, the complex mechanisms of existing antidepressant therapy along with poor prognosis aid in poor compliance. It is therefore need of the time to unveil alternative strategies to develop novel approaches for this purpose [7].

Neuroinflammation is involved in potentiating the severity of MDD, which is consistently reiterated in the literature [8, 9]. The surge in inflammatory mediators and cytokines cause the penetration of macrophages into the brain, validating the macrophage theory of depression [10]. Similarly, other research studies also implicated the role of inflammatory cascades in the pathophysiology of depression in both laboratory animals and meta-analysis of postmortem brain tissue samples [11, 12]. Furthermore, treatment with conventional antidepressants such as selective serotonin reuptake inhibitors (SSRIs) can reverse the elevated level of cytokine in addition to favorable outcomes on depression [13, 14]. However, other non-SSRIs can be used for the management of depression with no impact on cytokines [15]. This discrepancy is attributed to the heterogenetic nature of depressive disorders as MDD triggers proinflammatory cytokines [16, 17]. Maes et al. described inflammation as vital in propagating depression pathogenesis [18] as inflammatory cytokines trigger behavioral and cognitive deficits [19, 20], impaired neurotransmitter metabolism, and decrease neuroplasticity [21, 22]. Furthermore, the administration of lipopolysaccharide (LPS) can induce behavioral alterations in animals similar to that in humans [23, 24]. Based on these shreds of evidence, we used a well-studied inflammation inducer, lipopolysaccharide (LPS) to induce neuroinflammation, neurodegeneration, and behavioral deficits and thereby use it as a model of anxiety and depression in rodents [25–27].

It is well known that the cellular defense mechanism of the body involves the endogenous transcription factor nuclear factor erythroid 2-related factor 2 (Nrf2) against inflammation and oxidative stress. Nrf2 and Nrf2-mediated phase-II antioxidant enzymes have been well studied for their therapeutic role in the treatment of various neuronal disorders [28]. Furthermore, the contribution of Nrf2 in inflammation or inflammation-induced disorders such as stroke and other disorders is well documented in previous studies [29–31]. Therefore, dysregulation of the Nrf2 signaling pathway may cause increased susceptibility of the tissue to detrimental effects of oxidative stress and inflammatory mediators [32, 33]. Moreover, several research bodies have reported the neurotherapeutic role of Nrf2 and its downstream signaling in animal models of various neurological disorders [34]. Previously, it has been demonstrated that Nrf2 plays a crucial role in the pathophysiology of depression via regulating oxidative stress and inflammatory processes [35, 36]. Hence, targeting Nrf2 might be considered one of the potential pharmacological approaches for the inquisition of depressive behaviors.

Recently, studies suggest that food and nutritional supplement can modulate depressive-like symptoms [37–41], further supported by human meta-analyses [42, 43]. In line with these studies, natural moieties based on their rich antioxidant potential are frequently investigated as these drugs have therapeutic potential against many stress mediators, including inflammatory factors and free radical species [44]. Carveol, essential oil has previously demonstrated antidiabetic potential possibly by attenuating oxidative stress [45]. Furthermore, carveol has shown neuroprotective potential in the ischemic brain injury model by ameliorating the infarction area by promoting the Nrf2 pathway [33]. Also, carveol also demonstrated attenuation of memory impairment and behavioral deficits in rodent model possibly by ameliorating oxidative stress [46]. In another study, Zhang et al. reviewed that carveol and similar other natural oils mitigate depression-like symptoms [47]. Recently, we demonstrated that carveol attenuated acetaminophen-induced liver toxicity by modulating Nrf2 cascade and inflammatory cytokines [48]. Taking into account the pharmacological value of natural essential oils and the search for alternate drug therapy for depressive behaviors, the current study was designed to investigate the potential role of carveol against LPS-induced behavioral deficits, neuroinflammatory signals, and neurodegeneration in an animal model of rodents. Herein, we for the first time showed that carveol mediates its antidepressant and anxiolytic effect by regulating Nrf2 and its downstream inflammatory cascades.

## 2. Material and Methods

### 2.1. Chemicals and Reagents

All the chemicals and drugs such as carveol catalog number (192384-10G), all-trans retinoic acid (ATRA) trichloroacetic acid (TCA), 5,5′-Dithio-bis-(2-nitrobenzoic acid) (DTNB), glutathione (GSH), 1-Chloro-2,4-dinitrobenzene (CDNP), LPS, N-(1-Naphthyl) ethylenediamine dihydrochloride, and trichloroacetic acid (TCA) were purchased from Sigma-Aldrich (St. Louis, MO, USA). ABC Kit and primary antibodies were purchased from Santa Cruz Biotechnology such as an anti-HO-1 monoclonal antibody (mouse source, SC-136960), anti-Nrf2 (rabbit polyclonal, SC-722), anti-p-JNK (mouse monoclonal, SC-6254), anti-Bcl-2 (mouse monoclonal, sc-7382), and anti-COX-2 (mouse monoclonal, SC-514489). The secondary antibody (ab-6789) was purchased from Abcam (UK). The ELISA kits for Nrf2 (Cat # SU-B30429) and p-NF-*κ*B (Cat # SUB28069) were purchased from China (Shanghai Yuchun Biotechnology), and HO-1 (Cat # E-EL-R0488) and TNF-*α* (Cat # E-EL-R0019) ELISA kits were purchased from Elabscience.

### 2.2. Animals and Drug Treatment

The male Sprague Dawley rats having average body weight ranging from 180 to 200 g were kept in a condition of a 12-hour light and dark cycle with access to water and food in the animal house facility. The animals were provided standard temperature and humidity according to the standard laboratory protocols, similar to the ARRIVE guidelines. All the experiments were performed according to the standard protocols, Riphah Institute of Pharmaceutical Sciences (RIPS), Islamabad (Reference No: REC/RIPS/2020/07). The animals were acclimatized with the animal house facility before experimental procedures. The body weights were measured throughout the experimental period. The animals were divided into two experimental groups (a total of 80 animals) as follows (Figure 1).

### 2.3. Experimental Cohort 1

The first cohort was used to determine the effective dose of carveol (*n* = 10 animals/group) and consisted of saline, LPS, two carveol treatment groups with LPS as carveol 20 mg/kg (CAR 20) and carveol 50 mg/kg (CAR 50), and fluoxetine (5 mg/kg) with LPS. Saline, carveol, and fluoxetine were administered for 5 days as a single intraperitoneal dose (i.p), while LPS was administered on the 3rd and 4th day of the regimen either as a single dose or after carveol at a dose of 1 mg/kg, i.p, and fluoxetine injection as our previously reported data [27].

### 2.4. Experimental Cohort 2

The second cohort was used to determine the Nrf2 role and included three subgroupings (*n* = 10/group): ATRA in combination with LPS, carveol in combination with the ATRA + LPS group, and fluoxetine in combination with ATRA + LPS. ATRA was injected at least 30 min before LPS (i.p.).

### 2.5. Behavioral Studies

A gap period of at least 2 days was mentioned between each behavioral study.

#### 2.5.1. Sucrose Splash Test (SST)

The measurements were performed according to a standardized protocol as previously discussed [27]. The SST test was performed by spraying sucrose, and the typical parameters were recorded for 5 min, including licking and scraping the body to wash away the solution.

#### 2.5.2. Elevated Plus-Maze (EPM) Test

The LPS-mediated anxiety was measured by an EPM test using a framework located about 50 cm above the floor. The EPM test was performed by keeping each rat in the middle of the platform, and the number of entries and time spent was recorded [49].

#### 2.5.3. Light-Dark Box (LDB) Test

For the evaluation of anxiety-like behavior, the LDB test was performed using the customized light-dark box. The LDB is composed of light and dark compartments partitioned by a small gap or entry point. The test was performed by placing each experimental animal in the dark compartment of the light-dark box and was allowed to move freely in the box for 5 min. The data was recorded (videotaped), and the total number of entries in each compartment was noted. After completion of each test, the box was cleaned using alcohol to minimize the olfactory cues [50].

#### 2.5.4. Forced Swim Test (FST)

The forced swim test was performed to evaluate the depression level in rats. The rat was placed in a Plexiglas cylinder which was 70 cm in height and 30 cm in diameter, at a specific temperature of 23 ± 1°C. A preswim exposure test was performed 24 h before the test to delineate the antidepressant-like activity. The use of a preswim ensures that the rats quickly adopt an immobile posture on the test day, which enables the effect of the tested compounds to be more easily observed. The test was performed by filling the cylinder with water (above 30 cm height) at 23 ± 1°C temperature and videotaped for 7 min. The final 4 min time of the test was randomly assessed at 5 s intervals for various parameters such as immobility.

### 2.6. Antioxidant Assays

#### 2.6.1. Determination of Lipid Peroxidation (LPO)

This assay was performed according to our previously established laboratory protocol [51]. The tissue was homogenized in lysis buffer. The tissue homogenate was centrifuged, and the supernatant was further mixed with freshly prepared ammonium sulphate solution. After the addition of TBA, the absorbance was recorded at 532 nm.

#### 2.6.2. Reduced Glutathione (GSH) Level

The GSH assay was performed as previously described [52]. The 5,5′-Dithiobis-2-nitrobenzoic acid (DTNB) 0.6 mM was added to the 6.6 *μ*L sample, and the GSH level was measured as described previously [52]. The absorbance was recorded at 412 (nm) wavelength using a microplate reader.

#### 2.6.3. Glutathione S-Transferase (GST) Activity

The GST assay was performed for the activity of GST using the 1-Chloro-2,4-dinitrobenzene (CDNB) as a substrate as previously reported [53]. The assay protocol includes that each well was filled with 10 *μ*L of 1 mM CDNB, 10 *μ*L of 5 mM reduced glutathione, 270 *μ*L of buffer solution, and 10 *μ*L of the sample. The absorbance was read at 340 nm using a plate reader.

#### 2.6.4. Catalase Activity

The catalase assay was performed by mixing H_2_O_2_ and the tissue supernatant. The absorbance was measured at 240 nm wavelength compared with the blank containing PBS only. The absorbance or catalase activity is proportional to the degradation of H_2_O_2_ to its desired product. So actually, the assay determines the breakdown of H_2_O_2_ so the results are expressed as *μ*mol H_2_O_2_ decomposed per mg of protein/min [54].

### 2.7. Histological Preparation

The rats after behavioral analysis were decapitated, and the brain was removed. The brain was fixed, and the blocks were made. After that, we made three mm thick sections using a sharp blade and fixed in a 4% paraformaldehyde solution. The tissues were embedded into paraffin blocks and trimmed to 4 *μ*m thin coronal sections using a microtome, and the following staining techniques were applied.

### 2.8. Hematoxylin and Eosin (H&E) Staining

Starting from dewaxing/deparaffinization and then rehydration step using a gradient alcohol series, which was ended by rinsing slides in distilled water, slides were stained with hematoxylin and eosin as discussed [55]. Finally, slides were dehydrated, and color was fixed in xylene and observed by a light microscope (Olympus, Japan).

### 2.9. Immunohistochemical Analysis

We employed a previously described procedure with slight modifications for immunohistochemical analysis [56]. After completion of the deparaffinization step, slides were processed by an enzymatic method for antigen retrieval and then washed with PBS consecutively three times for 5 min. Slides were immersed in 3% H_2_O_2_ to quench endogenous peroxidase activity followed by washing with PBS. Normal goat serum (5%) was applied as a blocking serum, and slides were incubated for 2 h. Next, the slides were incubated overnight with primary antibodies Bcl2, p-JNK, TNF-*α*, Nrf2, HO-1, and COX-2. The next morning, slides were washed with PBS and incubated for 90 min with the secondary antibody, then incubated with an ABC kit (Santa Cruz) in a humidified box for 60 min. Slides were then washed with PBS solution and stained with DAB, followed by dehydration with ethanol (70%, 80%, 90%, and 100%). After dehydration, slides were fixed with xylene and then cover slipped with mounting media. Images were obtained using a light microscope and saved in TIFF format for further quantification by the ImageJ software.

### 2.10. ELISA Analysis

50-70 mg of cortical and hippocampal brain tissue was first homogenized and then centrifuged at 15,000 rpm at 4°C to carefully collect the supernatant while avoiding the pellet. ELISA procedures were performed according to the manufacturer protocols using an ELISA microplate reader (BioTek ELx808), and the concentration (pg/mL) was then normalized to the total protein content (pg/mg total protein).

### 2.11. Real-Time Polymerase Chain Reaction (RT-PCR)

Total RNA was extracted from the rat cortical tissue in TRIzol as discussed previously [57]. 20 *μ*L of M-MuLV reverse transcriptase was used to dilute 1 microgram of RNA and used this mix to synthesize cDNA with a cDNA synthesis kit (vivantis cDSK01-050 Sdn. Bhd, Malaysia). To estimate the gene expression of *Nrf2* quantitatively, real-time PCR was performed using the 2X HOT SYBR Green qPCR master mix (Solar Bio cat # SR1110) and real-time Mic PCR (BioMolecular System) according to the manufacturer specifications. The sequence of the primers used for amplification was *Nrf2*, Forward: CACATCCAGACAGACACCAGT and Reverse: CTACAAATGGGAATGTCTCTGC; *HO-1*, Forward: CGTGCAGAGAATTCTGAGTTC and Reverse AGACGCTTTACGTAGTGCTG; and GAPDH, Forward: AGGTCGGTGTGAACGGATTTG and Reverse: TGTAGACCATGTAGTTGAGGTCA. The relative gene expressions of *Nrf2* were determined by the 2^-*ΔΔ*CT method for real-time quantitative PCR.

### 2.12. Statistical Analysis

Data were analyzed using GraphPad Prism and were expressed as mean ± standard error of the mean (SEM). Data were further analyzed by one-way ANOVA while using post hoc as Bonferroni multiple comparisons. *p* < 0.05 was considered significant. The symbol ∗ shows a significant difference relative to the saline group, and # shows a significant difference relative to the LPS group, while † represents a significant difference to ATRA + LPS.

## 3. Results

### 3.1. Carveol Attenuated LPS-Induced Depression-Like Behavior

LPS-treatment induced depression-like behavior as shown by reduced struggling and by immobile nature in the behavioral FST (Figure 2(a), ∗∗*p* < 0.01), coexisting with anxiety-like behavior as entries to the open arms were little or absent in the EPM test and also the time spent in the open arms was short suggesting less exploration compared to the control group (Figure 2(b), ∗∗*p* < 0.01). In accordance, LPS caused a greater stay in the dark compartment in the LDB test (Figure 2(c), ∗∗∗*p* < 0.001), while significantly decreased grooming time in SST (Figure 2(d), ∗∗∗*p* < 0.001). Carveol treatment with 20 mg/kg dose reversed all these behavioral alterations in the FST (Figure 2(a), ^#^*p* < 0.05) and in the EPM test (Figure 2(b), ^#^*p* < 0.05), increased time spent in light compartment in LDB (Figure 2(c), ^#^*p* < 0.05), and increased the grooming time (Figure 2(d), ^#^*p* < 0.05) in SST. Similarly, treatment with carveol (50 mg/kg) produces the same effects in all these behavioral sets. Furthermore, cotreatment of LPS with ATRA exacerbated the anxiety-like behavioral deficits, while administration of carveol in this second cohort study did not elicit any ameliorative effects on LPS-induced depression-like behavior in the ATRA-treated groups.

### 3.2. Carveol Reversed LPS-Induced Cellular Damage

We performed HE staining to determine the rate and extent of neuronal cell death in response to LPS treatment, and we observed significant variations in neuronal shape and size (∗∗∗*p* < 0.001, Figure 3), compared to the saline group. The saline group exhibited normal morphological architecture of cell shape with no change in color staining, and there was no vacuole formation (Figure 3). Moreover, multiple vacuoles were noted in the LPS-treated groups associated with inflammatory infiltrated cells. Carveol administration mitigated these changes, and a higher degree of cellular integrity was evident in the carveol- (20 mg/kg-) treated group (Figure 3, ^##^*p* < 0.01). Furthermore, coadministration of LPS and ATRA exacerbated the histopathological changes while pretreatment of carveol in the ATRA-treated groups did not show any significant alteration in the LPS-induced histopathological changes.

### 3.3. Carveol Attenuated LPS-Induced Apoptosis Markers

To further evaluate the antiapoptotic properties of carveol, we performed immunohistochemistry analysis for antiapoptotic factor Bcl-2 and apoptosis-linked p-JNK (Figure 4(a)). The expression of the Bcl-2 protein was decreased (Figure 4(a), ∗∗*p* < 0.01), coexisting with an upregulated p-JNK level in the LPS-treated group (Figure 4(b), ∗∗*p* < 0.01). However, treatment with carveol reverts these changes in the LPS group. Moreover, carveol pretreatment did not attenuate the LPS-induced apoptosis in the cortex of the ATRA-treated groups.

### 3.4. Carveol Augmented the Antioxidant Potential of the Brain by Promoting the *Nrf2* Signaling Pathway

The mechanism of antioxidant capacity of carveol was determined by investigating the *Nrf2 gene* and Nrf2 protein and its downstream signaling *HO-1* gene and protein. Real-time PCR analysis showed that LPS treatment significantly reduced the expression level of *Nrf2* and *HO-1* compared to that of the control group (Figure 5(a), ∗*p* < 0.05). To further validate, we performed ELISA (Figure 5(b), ∗*p* < 0.05) and immunohistochemistry analysis (Figure 5(c), ∗∗*p* < 0.01), and consistent results were obtained. Likely, the downregulated proteins of Nrf2, antioxidant protein HO-1 expression was also significantly attenuated in the cortex and hippocampus of the LPS-treated group compared to that of the saline group (Figures 5(d)–5(f)). Administration of carveol along with LPS, induced upregulation of *Nrf2* and *HO-1* genes relative to that of the LPS group (Figures 5(a) and 5(d), ^##^*p* < 0.01). Furthermore, noticeably elevated levels of Nrf2 and HO-1 were also observed using ELISA and immunohistochemistry (Figures 5(b), 5(c), 5(e), and 5(f)). However, the carveol-mediated upregulation of the antioxidant proteins Nrf2 or HO-1 was not observed in the ATRA-treated groups. These results suggest that carveol might possess potential antioxidant activity via activation of the Nrf2 and its downstream proteins like HO-1.

### 3.5. Carveol Inhibits LPS-Induced Neuroinflammation

The role of inflammatory mediators in depression studies is well documented; therefore, we also sought to investigate whether carveol treatment can be effective against neuroinflammation. We studied the protein expression of inflammatory markers such as p-NFkB, COX-2, and TNF-*α* using ELISA and immunohistochemistry analysis. Our results showed that the levels of p-NFkB, TNF-*α*, and COX-2 were significantly increased in the LPS group compared to that of the saline group (Figures 6(a)–6(c)). Pretreatment of carveol induced a marked downregulation of p-NFkB (Figure 6(a), ^#^*p* < 0.05) and TNF-*α* (Figure 6(b), ^#^*p* < 0.05) in the cortex and COX-2 (Figure 6(c), ^#^*p* < 0.05 and ^##^*p* < 0.01) in the cortex and hippocampus relative to the LPS-treated group. Furthermore, cotreatment of LPS with ATRA further exaggerated the level of neuroinflammatory mediators, while carveol administration to the LPS- and ATRA-treated group did not show any protective effect against the detrimental effects of LPS and ATRA treatment.

### 3.6. Effects of Carveol Pretreatment on LPS-Induced Lipid Peroxidation and Antioxidant Enzymes

To investigate the neuroprotective and antioxidant activity of carveol, we measured the levels of various enzymes such as catalase, GST, GSH, and thiobarbituric acid reactive substances (TBARS) in both the cortex and hippocampus. Our results showed that carveol administration significantly ameliorated the LPS-induced oxidative stress via restoring the expression of the antioxidant enzymes in both the cortex and hippocampus. The levels of catalase, GST, and GSH were significantly lowered in the LPS-treated group compared to that of the saline group (Figures 7(a)–7(f), ∗∗∗*p* < 0.001 and ∗∗*p* < 0.01). In accordance, a marked elevation in the level of TBARS was observed in the LPS-treated brain compared to that of the saline group (Figures 7(g) and 7(h), ∗∗*p* < 0.01). Carveol administration induced the production of the antioxidant enzymes, i.e., catalase, GST, and GSH, in both the prefrontal cortex and hippocampus (Figures 7(a) and 7(b), ^##^*p* < 0.01; Figures 7(c) and 7(d), ^#^*p* < 0.05 and Figures 7(e) and 7(f), ^#^*p* < 0.05). On the other hand, a noticeably decreased level of TBARS was observed in the carveol-treated group as compared to that of the LPS-treated group (Figures 7(g) and 7(h), #*p* < 0.05). Furthermore, carveol administration in the ATRA-treated groups did not show any antioxidant activity (Figure 7), validating the results of endogenous antioxidant enzyme Nrf2 (Figure 5). Finally, our results revealed that carveol might possess potential free radical scavenging activity to attenuate the LPS-induced oxidative stress in the cortex and hippocampus of a rat's brain.

## 4. Discussion

Research studies in the recent decade have highlighted the role of phytochemicals in maintaining the brain's chemical balance and providing a potential source of neuroprotectants in several neurodegenerative diseases [58]. The goal of the present research study was to reveal the neurotherapeutic potential of the natural product, carveol against LPS-induced depression and anxiety in the rodent model. Carveol was used in this study based on its reported anti-inflammatory, antioxidant, anti-Alzheimer, and other neuroprotective properties [46, 59].

Accumulating evidence has shown that peripheral immune activation and increased cytokine production contribute to the development of depression [60]. LPS administration in rodents induces depressive and anxiety-like behaviors in several ways that include reduced locomotor activity and a decrease in struggling time in an unfavorable environment such as FST [61]. Here, in this study, we have shown that carveol pretreatment significantly attenuated the LPS-induced behavioral despair by increasing mobility and struggling time. Previous research studies have reported that decreased locomotor activity in the FST may be caused by the increased level of proinflammatory cytokines and reactive oxygen species (ROS) in the LPS model [61]. In accordance with previous studies, our results showed that carveol (20 mg/kg) mitigated depression-like symptoms induced by LPS. In addition to FST, we determined the grooming behavior of experimental rats in the SST, which may indicate decreased motivation and apathy. Our results pointed out that LPS administration significantly decreases the grooming time, hence inducing apathy and lack of motivation. Administration of carveol improved the core symptoms of depressive-like behaviors by mitigating LPS-induced behavioral despair and apathy. Furthermore, we also investigated anxiety-like behaviors by EPM and LDB tests. The data obtained from these paradigms determined the anxiolytic potential of carveol, as elevated values were observed in the open arm and lightbox parameters that indicate potential anxiolytic activity [62].

Several research bodies have demonstrated the involvement of oxidative stress and ROS in the pathophysiology of various neurological disorders [63, 64] including depression [65]. Our results attest to the previously reported data, that LPS administration induces an imbalance between endogenous antioxidant substances and stress agents, thereby stimulating the production of ROS and activation of the neuroinflammatory cascade. Furthermore, currently, several clinically used antidepressant drugs have potential ROS ameliorating effects in depressed patients. Among the various neuroinflammatory mechanisms, the *Nrf2* gene has been demonstrated as one of the major regulators of the cellular antioxidant system which involves transcription factor *Nrf2* and its downstream signalling protein HO-1 which modulates several anti-inflammatory and antioxidants genes [66]. Modulation of the Nrf2 pathway has been reported to play a major role in developing new strategies for neuronal protection [67]. Furthermore, the antidepressive activity of many protective agents has shown the upregulation of Nrf2 protein and its downstream signalling HO-1 in depression models [68]. Interestingly, our results are in line with previous studies indicating that the carveol-treated group reversed the LPS-induced increased levels of ROS and LPO and induces Nrf2/HO-1. These results validated our hypothesis that carveol may contain antioxidant potential and free-radical scavenging activity. To determine the possible mechanism for carveol-mediated neuroprotection, carveol along with ATRA (Nrf2 inhibitor) was administered to the LPS-intoxicated rats. Our results showed that inhibition of Nrf2 and HO-1 signalling pathways by ATRA treatment reversed the potential neuroprotective effects of carveol. Similarly, the biochemical assays also showed a significant decrease in levels of antioxidant enzymes (GSH, GST, and catalase) along with an increase in LPO and ROS levels in the ATRA-treated groups. This implies that Nrf2/HO-1 signalling pathway is a potential target in the antidepressant and anxiolytic activity of carveol. In accordance, our previous studies demonstrated that Nrf2 inhibition by ATRA increased infarction area in the MCAO model of ischemic stroke in rats [33]. Martín-de-Saavedra et al. stated that Nrf2 affects the monoamine mechanism of depression by modulating the level of different neurotransmitters such as dopamine, noradrenaline, and serotonin [36]. Furthermore, *Nrf2* knockout mice showed an increased level of glutamate accompanied by a significant decrease in the level of these neurotransmitters [36]. In addition, behavioral analysis in other research studies has shown an increase in immobility time in FST and a decrease in grooming time in SST in *Nrf2* null mice which further supports the role of Nrf-2 antagonism in depression [69]. It is well known that Nrf2 activation leads to the inhibition of inflammatory mediators via downregulating the NF-*κ*B signaling pathway. HO-1, downstream of Nrf2 is also known to be a potent inhibitor of proinflammatory cytokines [70, 71]. Consistent with previous research studies, our findings demonstrated that carveol effectively reversed the LPS-induced protein expression of various inflammatory mediators such as p-NFkB, TNF-*α*, and COX-2. Similarly, carveol upregulated the LPS-induced decreased protein expression of the antioxidant enzymes HO-1. Mechanistically, both the anti-inflammatory and antioxidant activities of carveol were diminished in the ATRA-treated groups, which supports our hypothesis that carveol exerts its protective activity via activating the Nrf2/HO-1 signaling pathway [71, 72].

Several lines of evidence have reported the involvement of MAP kinases such as JNK signaling in the induction of neuroinflammation-induced neurodegenerative disorders. Activation of the JNK also interferes with the BCL-2 family of proteins to induce cell death via activation of the mitochondrial apoptotic pathway [73]. In accordance, other studies have demonstrated a close interplay of JNK and caspase-3 in the apoptotic cascade [74, 75]. Our results demonstrated that carveol alleviated LPS-induced elevated levels of proapoptotic proteins and p-JNK.

## 5. Conclusion

Taken together, we can conclude from our results that carveol possesses potential antioxidant, anti-inflammatory, and neuroprotective properties. Further, our proposed neuroprotective mechanism suggests that carveol activated the endogenous antioxidant proteins like Nrf2 and HO-1 coupled to the downregulation of anti-inflammatory proteins like p-NF*κ*B and p-JNK. Collectively, these protective properties of carveol may offer a new therapeutic option for protecting the brain from neuroinflammation and oxidative stress.

## Figures and Tables

**Figure 1:** Experimental outline.

**Figure 2:** Effects of carveol (CAR) on LPS-induced behavioral deficits. Effect of CAR and LPS on the FST test (a), EPM (b), LDB (c), and SST (d). Data are expressed as means ± SEM and analyzed by one-way ANOVA followed by Bonferroni multiple comparisons test using the GraphPad Prism 6 software. The saline, LPS, CAR+LPS, and FLX + LPS groups represent the first cohort (*n* = 10/group), while the ATRA+LPS, CAR+ATRA+LPS, and ATRA+LPS + FLX were from the second cohort (*n* = 10/group). ^∗∗^*p* < 0.01 and ^∗∗∗^*p* < 0.01 are compared to the saline group; *^##^p* < 0.01 and #*p* < 0.05 indicate a significant difference compared to the LPS group. ^†^*p* < 0.05 is compared to ATRA+LPS. CAR: carveol; LPS: lipopolysaccharide; ATRA: all-trans retinoic acid; FLX: fluoxetine; EPM: elevated plus maze; FST: forced swim test; LDB: light-dark box; SST: sucrose splash test.

**Figure 3:** Hematoxylin and eosin (H&E) staining showing the extent of surviving neurons in the cortex and hippocampus (*Corno amonus*, *CA*). Scale bar 50 *μ*m, magnification 40x. Dead neurons were characterized by a swollen cytoplasm, vacuolization, scalloped morphology with intense cytoplasmic eosinophilia, and nuclear basophilia. Data are expressed as means ± SEM. ^∗∗∗^*p* < 0.001 is compared to the saline group; *^##^p* < 0.01 and #*p* < 0.05 indicate a significant difference compared to the LPS group; ^†^*p* < 0.05 is compared to ATRA+LPS. CAR 20: carveol (20 mg/kg); LPS: lipopolysaccharide; ATRA: all-trans retinoic acid; FLX: fluoxetine. The H&E slides were made after the euthanization of animals following behavioral analysis. The saline, LPS, CAR+LPS, and FLX + LPS groups were those studied in the first cohort (*n* = 5/group), while the ATRA+LPS, CAR+ATRA+LPS, and ATRA+LPS + FLX groups were from the second cohort (*n* = 5/group).

**Figure 4:** Effects of carveol on LPS-induced neuronal apoptosis. (a) Immunohistochemistry results for Bcl-2 in the cortex and hippocampus. Scale bar 50 *μ*m, magnification 40x. Data are expressed as means ± SEM. ^∗∗∗^*p* < 0.001 and ^∗∗^*p* < 0.01 are compared to the saline group; ##*p* < 0.01 and #*p* < 0.05 indicate a significant difference compared to the LPS group, while ^†^*p* < 0.05 is compared to ATRA+LPS. (b) Immunohistochemistry results for p-JNK in the cortex and hippocampus. Scale bar 50 *μ*m, magnification 40x. Data are expressed as means ± SEM. ^∗∗∗^*p* < 0.001 and ^∗∗^*p* < 0.01 are compared to the saline group; ##*p* < 0.01 and #*p* < 0.05 indicate a significant difference compared to the LPS group; †*p* < 0.05 is compared to ATRA+LPS. The immunohistochemistry sections were prepared after the euthanization of animals following behavioral analysis. The saline, LPS, CAR+LPS, and FLX + LPS groups were taken as the first cohort (*n* = 5/group), while the ATRA+LPS, CAR+ATRA+LPS, and ATRA+LPS + FLX groups were from the second cohort (*n* = 5/group). LPS: lipopolysaccharide; ATRA: all-trans retinoic acid; FLX: fluoxetine; p-JNK: Jun N-terminal kinase; Bcl-2: B cell lymphoma-2.

**Figure 5:** Effects of carveol on LPS-induced downregulation of *Nrf2* and *HO-1*. (a) RT-PCR analysis of *Nrf2* in the cortex. (b) Nrf2 protein level was measured by ELISA in the cortex and hippocampus. (c) Immunohistochemistry analysis of Nrf2 in cortex and hippocampus. Data are expressed as means ± SEM. ^∗∗^*p* < 0.01 and ^∗^*p* < 0.05 are compared to the saline group; ##*p* < 0.01 and #*p* < 0.05 indicate a significant difference compared to the LPS group, while ^†^*p* < 0.05 is compared to ATRA+LPS. A thick black arrow indicates nuclear localization of Nrf2 (d) RT-PCR analysis of *HO-1* in the cortex. (e) HO-1 protein level was measured by ELISA in the cortex and hippocampus. (f) Immunohistochemistry analysis of HO-1 in cortex and hippocampus. Data are expressed as means ± SEM. ^∗∗^*p* < 0.01 and ^∗^*p* < 0.05 are compared to the saline group; ##*p* < 0.01 and #*p* < 0.05 indicate a significant difference compared to the LPS group, while †*p* < 0.05 is compared to ATRA+LPS. The saline, LPS, CAR+LPS, and FLX + LPS groups were those studied in the first cohort (*n* = 5/group), while the ATRA+LPS, CAR+ATRA+LPS, and ATRA+LPS+ FLX groups were from the second cohort (*n* = 5/group). CAR 20: carveol (20 mg/kg); LPS: lipopolysaccharide; ATRA: all-trans retinoic acid; FLX: fluoxetine; *Nrf2*: nuclear factor E2-related factor; *HO-1*: heme oxygenase 1.

**Figure 6:** Effects of carveol on LPS-induced neuroinflammation. (a) p-NFKB and (b) TNF-*α* levels were measured by ELISA. Data are expressed as means ± SEM. (c) Immunohistochemistry results for COX-2 in the cortex and hippocampus. Scale bar 50 *μ*m, magnification 40x. Data are expressed as means ± SEM. ^∗^*p* < 0.05 and ^∗∗∗^*p* < 0.001 are compared to the saline group; ##*p* < 0.001 and #*p* < 0.05 indicate a significant difference compared to the LPS group, and †*p* < 0.05 is compared to ATRA+LPS. The saline, LPS, CAR+LPS, and FLX + LPS groups were those studied in the first cohort (*n* = 5/group), while the ATRA+LPS, CAR+ATRA+LPS, and ATRA+LPS+ FLX groups were from the second cohort (*n* = 5/group). CAR 20: carveol (20 mg/kg); LPS: lipopolysaccharide; ATRA: all-trans retinoic acid; FLX: fluoxetine; TNF-*α*: tumor necrosis factor-alpha; COX-2: cycloxygenase-2; p-NFkB: nuclear factor-kappa B.

**Figure 7:** Effects of carveol pretreatment on antioxidant enzymes and LPS-induced lipid peroxidation. Effects of LPS and CAR on levels of GSH (a, b), GST (c, d), catalase (e, f), and TBARS (g, h). Data are expressed as means ± SEM. ^∗∗^*p* < 0.01 and ^∗∗∗^*p* < 0.001 are compared to the saline group; ##*p* < 0.001 and #*p* < 0.05 indicate a significant difference compared to the LPS group, and †*p* < 0.05 or ††*p* < 0.01 is compared to ATRA+LPS. The saline, LPS, CAR+LPS, and FLX + LPS groups were those studied in the first cohort (*n* = 5/group), while the ATRA+LPS, CAR+ATRA+LPS, and ATRA+LPS+ FLX groups were from the second cohort (*n* = 5/group). CAR 20: carveol (20 mg/kg); LPS: lipopolysaccharide; ATRA: all-trans retinoic acid; FLX: fluoxetine; CAT: catalase; GSH: reduced glutathione; GST: glutathione S-transferase; TBARS: thiobarbituric acid reactive substances.

## Data Availability

The research data used to support the findings of this study are included within the article.
